The article "Possible Association Between COVID-19 Infection and De Novo Antineutrophil Cytoplasmic Antibody-Associated Vasculitis" was published in 2021. Journal: Cureus.

# Possible Association Between COVID-19 Infection and De Novo Antineutrophil Cytoplasmic Antibody-Associated Vasculitis

**DOI:** 10.7759/cureus.20331

**Published:** 2021-12-10

**Authors:** Nima Madanchi, Facundo E Stingo, Kennerly C Patrick, Selvaraj Muthusamy, Neha Gupta, Yahya Imran Fatani, Nehal Shah

**Affiliations:** 1 Rheumatology, Virginia Commonwealth University, Richmond, USA; 2 Pulmonary/Critical Care Medicine, Georgetown University/MedStar Washington Hospital Center, Washington D.C., USA; 3 Nephrology, Virginia Commonwealth University, Richmond, USA; 4 Renal Pathology, Virginia Commonwealth University, Richmond, USA; 5 Internal Medicine, Virginia Commonwealth University, Richmond, USA

**Keywords:** case report, pulmonary-renal syndrome, sars-cov-2, covid-19, anca-associated vasculitis

## Abstract

The coronavirus disease 2019 (COVID-19) has caused many different complications including immune-related conditions. Hereby, we report a case of a possible association between COVID-19 infection and de novo anti-neutrophil cytoplasmic antibodies (ANCA)-associated vasculitis presenting with severe pulmonary-renal syndrome as a rare complication of COVID-19 infection.

We had a 53-year-old male patient who was admitted for a severe COVID-19 pneumonia complicated by septic shock and acute respiratory distress syndrome. He responded to the standard treatments and was discharged. Four months later, he was admitted with a severe acute pulmonary-renal syndrome (severe acute on chronic kidney failure with active sediment and proteinuria, and diffuse alveolar hemorrhage (DAH) requiring mechanical ventilation). Kidney biopsy confirmed pauci-immune fibro-cellular crescentic glomerulonephritis on top of glomerular sclerosis. Perinuclear-ANCA and anti-myeloperoxidase antibody came back positive. Pulse steroids and cyclophosphamide were administered. Given the chronicity of the kidney lesions, the kidney function did not improve significantly, and the patient became dialysis dependent; however, respiratory status responded dramatically, and he was discharged on room air. In conclusion, although COVID-19 infection can mimic ANCA-associated vasculitis (AAV), the growing number of case reports along with our report shows the need for awareness of a potential link between COVID-19 infection and AAV which would dramatically change the treatment strategy.

## Introduction

The coronavirus disease 2019 (COVID-19) caused by the severe acute respiratory syndrome coronavirus-2 (SARS-CoV-2) has caused significant mortality and morbidity since its appearance in late 2019. COVID-19 has a strong link with thromboembolism [1], cardiomyopathy [2], and acute kidney injury (AKI) [3]. Lately, case reports have suggested an association between COVID-19, immune system dysregulation and cytokine storm. De novo presentation of anti-neutrophil cytoplasmic antibodies (ANCA)-associated vasculitis during COVID-19 has been recently reported in a few cases [4-11]. Patients presented with either AKI, diffuse alveolar hemorrhage (DAH), or both. Hereby, we present a case of newly diagnosed ANCA-associated vasculitis (AAV) in a patient with recent severe COVID-19 pneumonia who presented with both AKI and DAH.

The article "Possible Association Between COVID-19 Infection and De Novo Antineutrophil Cytoplasmic Antibody-Associated Vasculitis" was published in 2021. Journal: Cureus.

The case report’s abstract was previously presented as a virtual poster presentation at the 19th Annual Fellows Forum of The Rheumatism Society of the District of Columbia in May 2021.

## Case presentation

A 53-year-old incarcerated male with a past medical history of hypertension, hyperlipidemia, diabetes, chronic kidney disease stage 3, obstructive sleep apnea, latent tuberculosis, and previous transient ischemic attack, on aspirin, atorvastatin, insulin, metformin and hydrochlorothiazide on his baseline, tested positive for the SARS-CoV-2 virus at a correctional facility. After receiving an unknown treatment at this facility, he developed worsening hypoxia and was subsequently taken to our emergency department. He was initially treated with azithromycin and steroids, but the hospital course was complicated by septic shock and acute respiratory distress syndrome (ARDS) requiring intubation and mechanical ventilation. He was treated with convalescent plasma and broad-spectrum antibiotics. His hospital course was also complicated by AKI, and urinalysis was significant for hematuria, pyuria and sub-nephrotic range proteinuria. The AKI was not further evaluated as this injury was attributed to acute tubular necrosis in the setting of shock, and his kidney function improved during his hospitalization. Eventually, the patient's respiratory status improved; he was successfully extubated and discharged back to the correctional facility without the need for oxygen supplementation.

Four months later, the patient presented to a small community hospital with a one-week history of progressive dyspnea, chest pain and palpitations. In addition, he developed pink-tinged urine the day prior to the presentation. He was found to have new-onset atrial fibrillation with rapid ventricular response. He additionally had a hemoglobin of 6.6 g/dL, white blood cell (WBC) count of 13 x109/L, creatinine (Cr) of 8.7 mg/dL, blood urea nitrogen of 80 mg/dL, and bicarbonate 19 mEq/L. He was started on intravenous diltiazem drip for atrial fibrillation, given two units of red blood cells (RBCs), and single doses of ceftriaxone and azithromycin. He was then transferred to our hospital for further management.

The article "Possible Association Between COVID-19 Infection and De Novo Antineutrophil Cytoplasmic Antibody-Associated Vasculitis" was published in 2021. Journal: Cureus.

Upon arrival, he had a blood pressure of 170/123 mmHg, respiratory rate of 28 breaths per minute with an oxygen saturation of 96% on room air and was not febrile. He was in mild distress, had conjunctival pallor, crackles in bilateral bases, was in sinus rhythm with no murmurs, and had normal abdominal, neurologic, skin, and joint exam. Labs were significant for urine protein-to-Cr ratio of 2.2 mg/mg, and 5-10 of WBCs and RBCs per high powered field in the urinalysis. Urine microscopy was significant for numerous muddy brown casts with no cellular casts. C-reactive protein was 24.9 mg/dL and erythrocyte sedimentation rate was 87 mm/h. COVID-19 polymerase chain reaction was negative. Blood culture was negative. Chest computed tomography revealed bilateral patchy basilar opacities (Figure 1). Hospital course was complicated by shock requiring vasopressors, hypoxic respiratory failure requiring intubation and mechanical ventilation. Continuous renal replacement therapy was started for AKI. Given concern for vasculitis, he was started on pulse dose steroids. Bronchoscopy revealed bloody aspirate on multiple sampling but did eventually dilute, however, given worsening respiratory status, plasmapheresis was initiated. Bronchoalveolar lavage fluid was negative for infections. Perinuclear ANCA and anti-myeloperoxidase antibodies came back positive at 1:160 and 45 U/mL, respectively. Cytoplasmic and atypical ANCA, and anti-glomerular basement membrane antibody were negative. Kidney biopsy was performed, and microscopic examination showed 12-13 glomeruli of which two to six showed complete or near-complete glomerular sclerosis. Approximately three to four glomeruli showed cellular/early fibrocellular crescents. In addition, three to five glomeruli showed segmental scars. There was focal, active interstitial inflammation with focal lymphocytic tubulitis and mild atrophy and interstitial fibrosis.

**Figure 1:** Chest computed tomography of the patient on presentation

Immunofluorescence microscopy confirmed pauci-immune lesions consistent with AAV (Figures 2-4). Cyclophosphamide was given and steroids were tapered. The patient’s hemodynamics and oxygen requirement gradually improved. He was subsequently extubated and transitioned back to room air. He remained dialysis dependent throughout the hospitalization, and he was continued on hemodialysis at discharge to his correctional facility. Unfortunately, three months after discharge, he had not experienced recovery of kidney function and remained dependent on intermittent hemodialysis. He completed the course of treatment with cyclophosphamide infusions. During nine months of follow up till now, he has not had any flares and was started on azathioprine for maintenance.

The article "Possible Association Between COVID-19 Infection and De Novo Antineutrophil Cytoplasmic Antibody-Associated Vasculitis" was published in 2021. Journal: Cureus.

**Figure 2:** Cellular crescent on periodic acid-Schiff (PAS) stain

**Figure 3:** Fibrocellular crescent on periodic acid-Schiff (PAS) stain

**Figure 4:** Glomeruli with global sclerosis and fibrocellular crescent on trichrome stain

## Discussion

A series of recent publications have reported the development of vasculitis-like illness and auto-immune phenomena in patients recovering from COVID-19. The pathogenesis of the disease is still unknown; however, it is likely multifactorial. It has been described that during COVID-19 and its immediate recovery period, a robust activation of the immune system with the release of pro-inflammatory cytokines and immune system dysregulation/activation is present [12]. This was associated with an increased number of autoimmune conditions during this period, such as lymphocytic vasculitis, leukocytoclastic vasculitis, central nervous system vasculitis and Kawasaki disease, which are being increasingly reported [13]. Moreover, the disease in children has been associated with multi-system inflammatory syndrome either as a presenting syndrome or during recovery [7]. 

The association between COVID-19 and de novo AAV is rarer. To date, only a handful cases of possible association between COVID-19 and AAV have been reported. Patients have presented with either glomerulonephritis (GN), DAH, or both, during or shortly after COVID-19 [4-11]. This is a case report of a rare AAV presenting with pulmonary-renal syndrome in the immediate post infectious recovery. It is important to note that a causation cannot be proved, but an association is plausible. 

The pathogenesis of AAV-associated vasculitis has not been fully elucidated; however, it is thought to be multifactorial due to environmental factors in a patient with a genetic susceptibility, along with abnormalities in immune system regulation [14]. Both anti-myeloperoxidase and anti-proteinase-3 antibodies are strongly associated with AAV. Particularly in the case of COVID-19, the role of these antibodies has been explained with the evidence that neutrophil extracellular traps (NETs) as a source of autoantigens present myeloperoxidase and proteinase-3 to the immune system [4]. The presence of NETs has been observed on kidney biopsy samples of patients with AAV and is postulated to be involved in COVID-19 pathogenesis [4].

Another proposed hypothesis suggests that exposure to exogenous antigens can induce a pathogenic autoimmune response to the autoantigens resulting in AAV [15]. Furthermore, several infectious pathogens, such as Staphylococcus aureus and viruses, have been implicated in the pathogenesis of AAV [16]. Infectious pathogens may provide the initial antigen source to trigger innate and adaptive immune cell activation, thus signaling a pro-inflammatory state. As with most autoimmune diseases, genetically susceptible individuals are believed to experience a ‘second hit’ triggering an autoimmune response leading to AAV [15].

The article "Possible Association Between COVID-19 Infection and De Novo Antineutrophil Cytoplasmic Antibody-Associated Vasculitis" was published in 2021. Journal: Cureus.

Our patient presented with crescentic GN with severe AKI and DAH, which were diagnosed four months after recovering from severe COVID-19 pneumonia. Although the patient was found during his initial admission to have hematuria and proteinuria, they were believed not to be associated with AAV. There is strong evidence suggesting COVID-19 when presenting with ARDS can commonly cause AKI with proteinuria and hematuria [3,17]. The mechanism is believed to be an association of hemodynamic factors, viral tropism toward kidney tissue, and endothelial dysfunction leading to fibrinoid necrosis and development of microthrombi [18,19]. COVID-19 also commonly presents with significant air space disease in lung imaging which may look like DAH. Therefore, the clinical presentation of COVID-19 can mimic an AAV in many patients. Obviously differentiating these complications of COVID-19 from AAV would dramatically change the treatment strategy.

## Conclusions

As a rare manifestation, growing evidence is suggestive of a possible association between COVID-19 and AAV, although a causation cannot be proved. We encourage treating physicians to have a high clinical suspicion of de novo AAV in patients with active or recent SARS-CoV-2 infection when presenting with GN and/or DAH. 

## References

[1] Connors JM, Levy JH (2020). COVID-19 and its implications for thrombosis and anticoagulation. Blood.

[2] Tsao CW, Strom JB, Chang JD, Manning WJ (2020). COVID-19-associated stress (Takotsubo) cardiomyopathy. Circ Cardiovasc Imaging.

[3] Hirsch JS, Ng JH, Ross DW (2020). Acute kidney injury in patients hospitalized with COVID-19. Kidney Int.

[4] Uppal NN, Kello N, Shah HH (2020). De novo ANCA-associated vasculitis with glomerulonephritis in COVID-19. Kidney Int Rep.

[5] Hussein A, Al Khalil K, Bawazir YM (2020). Anti-neutrophilic cytoplasmic antibody (ANCA) Vasculitis presented as pulmonary hemorrhage in a positive COVID-19 patient: a case report. Cureus.

[6] Izci Duran T, Turkmen E, Dilek M, Sayarlioglu H, Arik N (2021). ANCA-associated vasculitis after COVID-19. Rheumatol Int.

[7] Reiff DD, Meyer CG, Marlin B, Mannion ML (2021). New onset ANCA-associated vasculitis in an adolescent during an acute COVID-19 infection: a case report. BMC Pediatr.

[8] Maritati F, Moretti MI, Nastasi V (2021). Anca-associated glomerulonephritis and anti-phospholipid syndrome in a patient with sars-cov-2 infection: just a coincidence?. Case Rep Nephrol Dial.

The article "Possible Association Between COVID-19 Infection and De Novo Antineutrophil Cytoplasmic Antibody-Associated Vasculitis" was published in 2021. Journal: Cureus.

[9] Moeinzadeh F, Dezfouli M, Naimi A, Shahidi S, Moradi H (2020). Newly diagnosed glomerulonephritis during COVID-19 infection undergoing immunosuppression therapy, a case report. Iran J Kidney Dis.

[10] Allena N, Patel J, Nader G, Patel M, Medvedovsky B (2021). A rare case of SARS-CoV-2-induced microscopic polyangiitis. Cureus.

[11] Powell WT, Campbell JA, Ross F, Peña Jiménez P, Rudzinski ER, Dickerson JA (2021). Acute ANCA vasculitis and asymptomatic COVID-19. Pediatrics.

[12] Dotan A, Muller S, Kanduc D, David P, Halpert G, Shoenfeld Y (2021). The SARS-CoV-2 as an instrumental trigger of autoimmunity. Autoimmun Rev.

[13] Becker RC (2020). COVID-19-associated vasculitis and vasculopathy. J Thromb Thrombolysis.

[14] Alba MA, Jennette JC, Falk RJ (2018). Pathogenesis of ANCA-associated pulmonary vasculitis. Semin Respir Crit Care Med.

[15] Xiao H, Hu P, Falk RJ, Jennette JC (2015). Overview of the Pathogenesis of ANCA-associated vasculitis. Kidney Dis.

[16] Popa ER, Tervaert JW (2003). The relation between Staphylococcus aureus and Wegener's granulomatosis: current knowledge and future directions. Intern Med.

[17] Kunutsor SK, Laukkanen JA (2020). Renal complications in COVID-19: a systematic review and meta-analysis. Ann Med.

[18] Ahmadian E, Hosseiniyan Khatibi SM, Razi Soofiyani S, Abediazar S, Shoja MM, Ardalan M, Zununi Vahed S (2021). Covid-19 and kidney injury: pathophysiology and molecular mechanisms. Rev Med Virol.

[19] Armaly Z, Kinaneh S, Skorecki K (2021). Renal manifestations of COVID-19: physiology and pathophysiology. J Clin Med.

